The article "Curcumin Prevents Diabetic Osteoporosis through Promoting Osteogenesis and Angiogenesis Coupling via NF-κB Signaling" was published in 2022. Journal: Evid Based Complement Alternat Med.

# Curcumin Prevents Diabetic Osteoporosis through Promoting Osteogenesis and Angiogenesis Coupling via NF-*κ*B Signaling

**DOI:** 10.1155/2022/4974343

**Published:** 2022-11-07

**Authors:** Desheng Fan, Jiuqing Lu, Nijia Yu, Yajia Xie, Lei Zhen

**Affiliations:** ^1^Department of Pathology, Baoshan Branch, Shuguang Hospital, Shanghai University of Traditional Chinese Medicine, Shanghai 201999, China; ^2^Oral Biomedical Engineering Laboratory, Shanghai Stomatological Hospital, Fudan University, Shanghai 200001, China; ^3^Department of Stomatology, Tongji Hospital, School of Medicine, Tongji University, Shanghai 200065, China

## Abstract

Diabetic osteoporosis (DOP) is a metabolic disease which is characterized by impaired bone microarchitecture and reduced bone mineral density resulting from hyperglycemia. Curcumin, an effective component extracted from *Curcuma longa*, exhibits antioxidation, regulation of bone metabolism and hypoglycemic effects. The BMSC-mediated osteogenesis and angiogenesis coupling seems to be important in bone formation and regeneration. We aimed to explore the effect of curcumin on BMSC-mediated osteogenesis-angiogenesis coupling in high glucose conditions and underlying mechanisms. Our results showed that high glucose impaired the osteogenic and proangiogenic ability of BMSCs and that curcumin pretreatment rescued the BMSC dysfunction induced by high-concentration glucose. Inhibition of the high glucose-activated NF-*κ*B signaling pathway has been found to contribute to the protective effects of curcumin on high glucose-inhibited coupling of osteogenesis and angiogenesis in BMSCs. Furthermore, accelerated bone loss and decreased type H vessels were observed in diabetic osteoporosis mice models. However, curcumin treatment prevented bone loss and promoted vessel formation in diabetic osteoporosis mice. Based on these results, we concluded that curcumin ameliorated diabetic osteoporosis by recovering the osteogenesis and angiogenesis coupling of BMSCs in hyperglycemia, partly through inhibiting the high glucose-activated NF-*κ*B signaling pathway.

## 1. Introduction

Diabetic osteoporosis (DOP) is becoming an increasing complication of diabetes, which is characterized by destructive bone microarchitecture and reduced bone mineral density (BMD) [1–5]. Compared with normoglycemic individuals, patients with DOP have a significantly increased risk of fractures, leading to high disability and mortality rates [6, 7]. However, an ideal treatment for DOP is currently lacking.

Bone regeneration and remodeling are associated with the osteogenesis and angiogenesis coupling [8, 9]. Meanwhile, cross-talk between BMSCs and endothelial cells seems to be vital in bone regeneration [10–13]. Endothelial cells are largely dedicated to the improvement of the recruitment and osteogenic differentiation of BMSCs. Conversely, BMSCs secrete multiple proangiogenic growth factors to promote angiogenesis and tissue regeneration. However, much evidence has shown that the declined osteogenic differentiation function and angiogenesis ability of BMSCs is an important mechanism of DOP [14–17]. Therefore, restoring the damaged osteogenesis and angiogenesis function of BMSCs is crucial for the treatment of DOP.

The article "Curcumin Prevents Diabetic Osteoporosis through Promoting Osteogenesis and Angiogenesis Coupling via NF-κB Signaling" was published in 2022. Journal: Evid Based Complement Alternat Med.

Curcumin, an effective component extracted from *Curcuma longa,* exhibits antioxidation, regulation of bone metabolism, and hypoglycemic effects [18–26]. Reports demonstrate that curcumin may ameliorate bone microarchitecture and enhance BMD in APP/PS1 transgenic mice [27] and has shown bone protective effect on postmenopausal osteoporosis animal models and patients [28–32]. More importantly, recent studies have found the therapeutic value of curcumin on osteoporosis induced by diabetes [33, 34]. The benefits of curcumin on bone formation and regeneration are attributed to its capacity to reduce H_2_O_2_-stimulated osteoblast apoptosis [35], improving osteoblast mitochondrial function [36], and recovering the high glucose-impaired osteogenic differentiation of osteoblast and BMSCs [37, 38]. However, the effect of curcumin on BMSCs-mediated osteogenesis and angiogenesis coupling in high glucose microenvironments and the mechanisms underlying it are not clear.

NF-*κ*B, which is known as a master transcription factor, contributes to the development of diabetes and its complications. Inactivation of NF-*κ*B can reduce inflammatory cytokine secretion in diabetic animal models and patients [39, 40]. Furthermore, studies have discovered that NF-*κ*B signaling pathway have a significant influence on osteoporosis therapy and bone regeneration [41, 42]. Downregulation of NF-*κ*B p65 expression drastically alleviates osteoporosis in OVX mice [43]. The activated NF-*κ*B signaling pathway inhibits BMSCs mediation of the bone regeneration and angiogenesis in a distraction osteogenesis model [44]. Hence, these findings demonstrate that inhibiting overactivated NF-*κ*B pathway may be a new way for the treatment of diabetes and osteoporosis.

We aimed to investigate whether curcumin could rescue high glucose-inhibited osteogenesis and angiogenesis of BMSCs. In addition, we examined whether inhibiting overactivated NF-*κ*B signaling pathway contribute to the protective effects of curcumin on BMSCs dysfunction. Furthermore, we used a DOP model to explore the effects of curcumin on bone regeneration and vessel formation *in vivo*. The current study laid the foundation for curcumin in the treatment of DOP.

The article "Curcumin Prevents Diabetic Osteoporosis through Promoting Osteogenesis and Angiogenesis Coupling via NF-κB Signaling" was published in 2022. Journal: Evid Based Complement Alternat Med.

## 2. Materials and Methods

All animal protocols and experiments were approved by the Institutional Committee for Animal Use and Care at Shanghai University of Traditional Chinese Medicine.

### 2.1. Cell Cultures

C57BL/6 male mice of six-week-old (SLAC Laboratory Animal Co. Ltd., China) were used to obtain bone marrow samples. BMSCs were isolated from the bone marrow. The cells were inoculated in culture dishes containing DMEM (HyClone) and 10% FBS (Gibco). BMSCs from passages 2–4 were used in our study.

### 2.2. Cell Viability

BMSCs were treated with curcumin (Cur; Sigma-Aldrich) from 0.1 *μ*M to 10 *μ*M for 48 hours. After that, a CCK-8 kit was used to measure the cell viability.

### 2.3. BMSCs Osteogenic Differentiation

Cells were cultured with 5.5 mM glucose as the control group (NG), and BMSCs treated with 33 mM glucose represented the high glucose group (HG). For the curcumin groups, cells were cultured with 33 mM glucose and 1 *μ*M curcumin (HG + Cur). After seven days of osteogenic induction, ALP staining analysis and ALP activity was detected. After 21 days of culture, calcium nodules were detected through staining with a 2% alizarin red S solution (Solarbio, China).

### 2.4. Quantitative Real-Time PCR (qRT-PCR) Analysis

Total RNA was extracted using TRIzol reagent (Tiangen, China). One microgram of cDNA templates was used for qRT-PCR analysis. The expression of the mRNAs was calculated via the comparative cycle threshold method against GAPDH. The primers were as follows:

Runx2 F: 5′CTCAGCAGCAGCAGCAGCAG3′, R: 5′GCACGGAGCACAGGAAGTTGG3′; OCN F: 5′GAATCGGGGGATGTACCCAC3′, R: 5′CGAAGGCCTCTGGTTCCACT3′; OSX F: 5′GGATTGGATCTGAGTGAGCC3′, R: 5′GCCATAGTGAGCTTCTTCCTGG3′; VEGF F: 5′CGAGCAGCGAAAGCGACAGG3′, R: 5′CGAAGCGAGAACAGCCCAGAAG3′; GAPDH F: 5′GTCCATGCCATCACTGCCACTC3′, R: 5′CGCCTGCTTCACCACCTTCTT3′.

### 2.5. Conditioned Medium (CM) of BMSCs

After 48 hours of treatment with or without curcumin, BMSCs were cultured in fresh DMEM for an additional 48 hours. Then, the CM from each group (CM^NG^ group, CM^HG^ group, and CM^HG^ ^+^ ^Cur^ group) was harvested.

### 2.6. Enzyme-Linked Immunosorbent Assay (ELISA)

An ELISA kit (Beyotime Biotechnology, China) was used to detect the concentration of VEGF in different conditioned media.

### 2.7. EdU Analysis

HUVECs were cultured with different CM for 24 hours and incubated in EdU working solution (Beyotime Biotechnology, China) for 2 hours. After fixation for 15 minutes with 4% paraformaldehyde, cells were treated with the click additive solution for another 15 min. Finally, the nuclei were stained using a Hoechst solution.

The article "Curcumin Prevents Diabetic Osteoporosis through Promoting Osteogenesis and Angiogenesis Coupling via NF-κB Signaling" was published in 2022. Journal: Evid Based Complement Alternat Med.

### 2.8. Scratch Wound Assay

HUVECs were inoculated in six-well plates and grown to 100% confluence. Two parallel scratches were generated in each well using a 200 *μ*L pipette tip, and the medium was replaced with CM. After 24 hours, the scratched areas were measured.

### 2.9. Tube Formation

Cells were inoculated onto Matrigel-coated96-well plates and cultured with different CM for 24 hours. The tubule number and lengths were quantified using ImageJ software.

### 2.10. Immunofluorescence Staining

BMSCs were incubated with an anti-p65 antibody (1 : 200; Abcam, United Kingdom) at 4°C overnight and were treated with secondary antibody (1 : 500; Cell Signaling Technology) in the dark for another 1 hour.

### 2.11. Western Blot

Cells were lysed with RIPA lysis buffer for 30 min and proteins were extracted. Protein samples were electrophoresed on 5–12% SDS-polyacrylamide gels. The pretreated PVDF membrane (Invitrogen) was used to transfer the fractionated proteins. Then, the PVDF membrane was blocked for 1 hour and incubated with anti-p65 (1 : 1,000; Abcam), anti-phosphorylated p65 (p-p65; 1 : 500, Abcam), anti-Runx2 (1 : 1,000; Cell Signaling Technology), anti-VEGF (1 : 1,000; Cell Signaling Technology), anti-*β*-actin (1 : 2000; Cell Signaling Technology), anti-GAPDH (1 : 2,000; Cell Signaling Technology), and anti-LaminB (1 : 2,000; Cell Signaling Technology) primary antibodies overnight at 4°C. The membrane was incubated in the secondary antibodies (1 : 5,000; Invitrogen) for 1 hour.

### 2.12. Animals and Treatment

Fifteen six-week-old C57BL/6 male mice received intraperitoneal injections of streptozotocin (STZ, 50 mg/kg; Sigma-Aldrich) to induce DM. At three and seven days after STZ injection, the fasting blood glucose (FBG) was detected using a glucometer (OMRON, Japan). Only mice with FBG two times higher than 16.7 mmol/L were considered successful models of DM [45–48]. Twelve mice fit the criterion and were divided into two groups (*n* = 6 mice per group) according to the treatment: DM and DM + curcumin (DM + Cur). The other six mice were grouped into the control group. Curcumin was administered via gavage at a dose of 100 mg/kg/day for eight weeks after the establishment of the DM model.

### 2.13. Micro-CT Analysis

At the end of these experiments, the mouse femur samples were analyzed using a micro-CT system. The region of interest (ROI) was selected and the following parameters were calculated.

### 2.14. Microfil Perfusion

Cardiac Microfil (FlowTech) perfusion was performed to evaluate the neovascularization. Subsequently, the perfused mice were placed at 4°C for 24 h, and then the femur samples were decalcified for four weeks. The vessel formation were analyzed using a micro-CT system.

The article "Curcumin Prevents Diabetic Osteoporosis through Promoting Osteogenesis and Angiogenesis Coupling via NF-κB Signaling" was published in 2022. Journal: Evid Based Complement Alternat Med.

### 2.15. Immunofluorescence Staining of Bone Tissue

The sections were incubated with a CD31 antibody (1 : 100; Abcam) and an endomucin (EMCN) antibody (1 : 100; Santa Cruz) together at 4°C overnight and then were incubated with secondary antibodies (1 : 200; Santa Cruz) for 1 hour. The images were photographed with a camera. The CD31^hi^Emcn^hi^ type vessels were measured using Image-Pro Plus software based on color recognition.

### 2.16. Statistical Analysis

All experimental data are presented as mean ± SD and the statistical analysis was tested using Student's *t*-test and one-way ANOVA with SPSS 17.0 software.

## 3. Results

### 3.1. Curcumin Rescued the High Glucose-Inhibited BMSCs Osteogenic Differentiation

CCK-8 results showed that curcumin ranging from 0.1 *μ*M to 1 *μ*M was not significantly influenced on cell viability; however, 5 *μ*M and 10 *μ*M curcumin decreased cell viability (Figure 1(a)). Several studies have suggested that high concentrations of glucose can suppress the BMSCs osteogenic differentiation. We, therefore, determined whether curcumin could rescue the high glucose-induced osteogenic dysfunction of BMSCs *in vitro*. Our results demonstrated that curcumin pretreatment significantly reversed the decrease in ALP staining and activity induced by high glucose (Figure 1(b)). Similarly, alizarin red staining and semiquantitative analysis results also showed that the reduced mineralization nodule formation under high glucose conditions was recovered by curcumin (Figure 1(c)). Furthermore, the decreased mRNA and protein expression of osteogenic markers in high glucose conditions was recovered by curcumin administration (Figures 1(d)–1(f)). These findings revealed that curcumin promoted BMSCs osteogenic differentiation in high glucose.

### 3.2. Curcumin Recovered the High Glucose-Impaired Proangiogenic Ability of BMSCs

Based on the results of the EdU test, HUVECs cultured in CM^HG^ showed decreased proliferation compared with cells cultured with CM^NG^; however, CM^HG^ ^+^ ^Cur^ treatment significantly reversed the decrease in proliferation induced by CM^HG^ (Figures 2(a) and 2(b)). In addition, the migration capacity of HUVECs was suppressed after stimulation with CM^HG^, and the migration area was significantly increased in the CM^HG^ ^+^ ^Cur^ group compared with the CM^HG^ group (Figures 2(c) and 2(d)). Moreover, CM^HG^ markedly impaired the tube formation ability of HUVECs compared to that of the CM^NG^ group; however, CM^HG^ ^+^ ^Cur^ treatment significantly rescued the tube formation of HUVECs cultured with CM^HG^ (Figures 2(e)–2(g)).

### 3.3. Curcumin Promoted the Angiogenesis Potential of BMSCs by Increasing VEGF Expression and Secretion

In the present study, we observed markedly reduced VEGF protein expression in BMSCs exposed to HG compared with cells exposed to NG, whereas the HG-induced suppression of VEGF expression was reversed by curcumin (Figures 3(a) and 3(b)). Moreover, the production of VEGF in the CM from high glucose-induced BMSCs was much lower than that in the normal glucose group and that curcumin pretreatment increased the concentration of VEGF from high glucose + curcumin group (Figure 3(c)). To further investigate whether VEGF mediated curcumin-promoted angiogenesis in high glucose conditions, VEGF neutralizing antibodies were used. As shown in Figures 3(d)–3(j), blocking VEGF remarkably suppressed the curcumin-enhanced angiogenesis capacity of BMSCs in high glucose.

The article "Curcumin Prevents Diabetic Osteoporosis through Promoting Osteogenesis and Angiogenesis Coupling via NF-κB Signaling" was published in 2022. Journal: Evid Based Complement Alternat Med.

### 3.4. NF-*κ*B Signaling is Involved in the Effects of Curcumin on BMSCs-MediatedOsteogenesis-Angiogenesis Coupling

Western blot results showed that high-concentration glucose increased the phosphorylation levels of NF-*κ*B p65 (p-p65) without changing the total NF-*κ*B p65 levels (Figures 4(a) and 4(b)). However, curcumin decreased p-p65 levels promoted by high glucose (Figure 4(c)). In addition, high glucose upregulated the nuclear protein expression of NF-*κ*B p65 in BMSCs, whereas curcumin treatment attenuated nuclear NF-*κ*B p65 (Figure 4(d)). Immunofluorescence assays also found that the nuclear localization of the NF-*κ*B p65 protein in curcumin-treated cells was weaker than that in high glucose-stimulated cells (Figures 4(e) and 4(f)).

We subsequently explored whether the coupling of osteogenesis-angiogenesis in high glucose could be impacted by modulating NF-*κ*B signaling. Our results showed that cells cultured in high glucose supplemented with Bay117082, a specific NF-*κ*B inhibitor, exhibited decreased p-p65 activity compared with that of cells incubated with high glucose only (Figures 5(a) and 5(b)). However, ALP and alizarin red staining results showed that BMSCs treated with Bay117082 exhibited substantially higher levels of ALP activity and mineralization nodule formation than cells treated with high glucose (Figures 5(c) and 5(d)). Moreover, the suppressed migration and tube formation ability of HUVECs stimulated with CM^HG^ was reversed by treatment with CM^HG^ ^+^ ^Bay117082^ (Figures 5(e)–5(h)). We also observed that Bay117082 significantly upregulated osteogenesis and angiogenesis-related proteins Runx2 and VEGF expression (Figures 5(i) and 5(j)). All these data suggested that curcumin action on BMSCs-mediated osteogenesis-angiogenesis couples partly through the NF-*κ*B signaling pathway.

The article "Curcumin Prevents Diabetic Osteoporosis through Promoting Osteogenesis and Angiogenesis Coupling via NF-κB Signaling" was published in 2022. Journal: Evid Based Complement Alternat Med.

### 3.5. Curcumin Prevented Diabetes-Induced Bone Loss and Promoted Vessel Formation

The micro-CT results showed that curcumin treatment rescued the reductions of BV/TV, Tb. N, Tb. Th, and BMD in DM mice (Figures 6(b)–6(g)). The microfil showed a reduced vessel network in the DM group while more vessel formation was detected in the DM + curcumin group (Figure 6(h)). Furthermore, the role of curcumin in type *H* vessel was investigated. Immunofluorescence staining showed that curcumin administration increased the number of type *H* vessels in DM mice (Figures 6(i) and 6(j)). These results revealed that curcumin treatment prevented diabetes-induced bone loss and promoted vessel formation *in vivo*.

## 4. Discussion

Some studies have proven that osteogenesis and angiogenesis coupling plays a vital role in the pathogenic progression of DOP [14–17]. In the study, we demonstrated that curcumin treatment could enhance BMSC-mediated osteogenesis and angiogenesis coupling in high glucose microenvironments. Mechanistically, the effects of curcumin on BMSC osteogenic determination and BMSC-mediated angiogenesis were achieved, at least partially, by inhibiting the high glucose-activated NF-*κ*B signaling pathway. Furthermore, we confirmed that curcumin treatment promoted bone regeneration and accelerated angiogenesis in a DM model. To our knowledge, this is the first to confirm that curcumin prevents diabetes-induced bone loss by promoting BMSC-mediated osteogenesis and angiogenesis coupling.

BMSCs are a cell type which have self-renewal and multidirectional differentiation potential. It is well known that osteogenesis ability of BMSCs plays a crucial role in bone repair and regeneration. However, increasing evidence has shown that the decline in the osteogenic function of BMSCs is a vital mechanism for diabetic osteoporosis. BMSCs derived from diabetic patients show a decreased osteogenic differentiation ability [49]. In a high glucose microenvironment, advanced glycation end products (AGEs) induce Wnt/LRP5/*β*-catenin to inhibit the BMSCs osteogenic differentiation [50]. These studies suggest that hyperglycemia can lead to a change in BMSCs differentiation function, resulting in a decrease in the self-repair and regeneration ability of the bone tissue and related pathological changes in diabetic osteoporosis. Recently, an increasing number of reports have shown that curcumin possesses favorable properties on diabetic bone metabolism [32–34]. Li and Zhang founded that curcumin pretreatment could promote osteogenesis of BMSCs in high glucose and enhanced bone formation in diabetic rats by regulating the Keap1/Nrf2/HO-1 signaling pathway [3]. Another study showed that curcumin enhanced osteogenesis-related gene expressions and suppressed apoptosis in osteoblasts under high glucose microenvironment [35, 36]. In this study, our results showed that curcumin treatment rescued high glucose-inhibited osteogenic differentiation ability of BMSCs *in vitro*. Furthermore, our *in vivo* results also revealed that curcumin prevented bone loss in diabetic mice.

The article "Curcumin Prevents Diabetic Osteoporosis through Promoting Osteogenesis and Angiogenesis Coupling via NF-κB Signaling" was published in 2022. Journal: Evid Based Complement Alternat Med.

The osteogenesis and angiogenesis coupling is crucial in the process of bone regeneration. There is increasing evidence that BMSCs promote vessel formation in the skeletal system based on the coupling between osteogenesis and angiogenesis. BMSCs not only induce differentiation into endothelial cells to form vascular-like tissue but also produce multiple proangiogenic growth factors to promote angiogenesis [51, 52]. Moreover, the proangiogenic ability of BMSCs is regulated by many factors. Platelet-derived growth factor-B (PDGF-B) gene overexpression in BMSCs can enhance angiogenesis and promote the repair of bone defects [53]. BMSCs derived from OVX rats showed a decreased angiogenesis ability [11]. Catalpol, a natural iridoid glycoside, accelerates bone regeneration through improving the angiogenesis of BMSCs [13]. However, the influence of curcumin on the ability of BMSCs to regulate angiogenesis has been rarely reported. In this study, we verified that curcumin could rescue the high glucose-impaired angiogenic ability of BMSCs by elevating the expression and secretion of the proangiogenic factor VEGF. Besides, we proved that curcumin treatment promoted vessel formation in the DM model.

Recently, type *H* vessels were discovered in mouse and human bone tissues that is characterized by the high expression of CD31 and endomucin (CD31^hi^Emcn^hi^). Type H vessels secrete factors such as HIF-1*α*, VEGF, and Notch that promote vessel assembly and bone formation [16, 17]. Given the important role of type *H* vessels in coupling osteogenesis and angiogenesis, the effect of curcumin on type *H* vessels in DM mice was investigated. Our results showed a decreased number of type *H* vessels in DM mice, but curcumin administration increased the quantity of vessels.

Activation of the NF-*κ*B pathway is involved in diabetes and osteoporosis [38–40]. Inhibiting overactivated NF-*κ*B pathway promotes the differentiation and mineralization of MC3T3 cells [54]. NF-*κ*B inhibitor treatment rescues high glucose-dependent inflammatory cytokine expression and PDLSCs osteogenic differentiation [55, 56]. In this study, we found that the activated NF-*κ*B signaling pathway was inhibited by curcumin treatment in BMSCs. Moreover, Bay117082, an NF-*κ*B inhibitor, was used to investigate the role of NF-*κ*B in high glucose-induced BMSCs dysfunction. Our results showed that Bay117082 treatment reversed the glucose-inhibited osteoblastic differentiation and angiogenesis of BMSCs *in vitro*. Taken together, the above results indicated that curcumin rescued the high glucose-impaired osteogenesis and angiogenesis coupling of BMSCs via inhibiting the overactivated NF-*κ*B signaling pathway.

The article "Curcumin Prevents Diabetic Osteoporosis through Promoting Osteogenesis and Angiogenesis Coupling via NF-κB Signaling" was published in 2022. Journal: Evid Based Complement Alternat Med.

## 5. Conclusions

Our findings reveal the effects of curcumin in promoting the BMSCs-mediated osteogenesis and angiogenesis coupling in high glucose conditions. These impacts are preliminarily considered to be via NF-*κ*B signaling pathway inhibition. Furthermore, curcumin may become a potential drug to prevent and treat diabetic osteoporosis through promoting bone regeneration and vessel formation.

## Figures and Tables

**Figure 1:** Curcumin (Cur) rescued HG-induced osteogenic dysfunction of BMSCs. (a) Cell viability was determined by CCK-8 in the presence of different concentration of Cur for 24 h. (b)–(f) Osteogenic differentiation of BMSCs treated with Cur and different concentrations of glucose were determined with (b) ALP staining and ALP activity assays; (c) alizarin red staining and calcium deposition analysis; (d) expression of osteogenic-specific genes were assessed with qRT-PCR; (e)–(f) the expression of Runx2 by western blot. Data are presented as the mean ± SD from at least three independent experiments. ^Δ^*p* < 0.05, ^ΔΔ^*p* < 0.01, versus 0 *μ*M Cur group. ^*∗*^*p* < 0.05 and ^*∗∗*^*p* < 0.01 versus NG group. ^#^*p* < 0.05 and ^##^*p* < 0.01 versus HG group.

**Figure 2:** Cur recovered HG-impaired proangiogenic ability of BMSCs. Endothelial cells stimulated with conditioned medium (CM) from BMSCs treated with NG, HG, and HG + Cur. (a)–(b) Proliferation was determined by EDU555 staining. (c)–(d) Endothelial cell motility in each group was evaluated using the scratch wound assay. (e)–(g) Representative images (e) and quantification of tube formation (f)–(g) were assessed in each group. Data are presented as the mean ± SD from at least three independent experiments. ^*∗*^*p* < 0.05 and ^*∗∗*^*p* < 0.01 versus NG group. ^#^*p* < 0.05 and ^##^*p* < 0.01 versus HG group.

**Figure 3:** Cur increased VEGF expression and secretion to improve the proangiogenic capacity of BMSCs in HG. (a)–(b) VEGF protein expression of BMSCs in each group were assessed using western blot. (c) Detection of VEGF concentration in conditioned medium from BMSCs in each group using ELISA. (d)–(j) Endothelial cells were incubated with Cur pretreated BMSC CM, supplemented with or without VEGF neutralizing antibodies. (d)–(e) Proliferation was determined by EDU555 staining. (f)–(g) Cell motility in each group was evaluated using the scratch wound assay. (h)–(j) Representative images and quantification of tube formation were assessed in each group. Data are presented as the mean ± SD from at least three independent experiments. ^*∗*^*p* < 0.05 and ^*∗∗*^*p* < 0.01 versus NG group. ^#^*p* < 0.05 and ^##^*p* < 0.01 versus HG group. ^&^*p* < 0.05 and ^&&^*p* < 0.01 versus CMHG + Cur group.

The article "Curcumin Prevents Diabetic Osteoporosis through Promoting Osteogenesis and Angiogenesis Coupling via NF-κB Signaling" was published in 2022. Journal: Evid Based Complement Alternat Med.

**Figure 4:** Cur regulated NF-*κ*B signaling in BMSCs. (a)–(b) Western blot of p65 and p-p65 in BMSCs treated with NG and HG. (c) Western blot of p65 and p-p65 in BMSCs treated with NG, HG, and HG + Cur. (d) The nuclear protein levels of p65 were detected by western blot in NG, HG, and HG + Cur group. (e) BMSCs were fixed and incubated with an anti-p65 antibody. Nuclei were stained by DAPI. The nuclear and cytoplasm images were merged in the same visual field. (f) Quantitative analysis of the nuclear translocation of p65. Data are presented as the mean ± SD from at least three independent experiments. ^*∗*^*p* < 0.05 and ^*∗∗*^*p* < 0.01 versus NG group. ^#^*p* < 0.05 and ^##^*p* < 0.01 versus HG group.

**Figure 5:** NF-*κ*B signaling is involved in HG-inhibited osteogenic differentiation and proangiogenic ability of BMSCs. Western blot of p65 and p-p65 in BMSCs treated with HG or HG + Bay117082 (Bay) (a) and (b). Osteogenic differentiation of BMSCs treated with HG or HG + Bay were determined with (c) ALP staining and ALP activity assays, and (d) alizarin red staining and calcium deposition analysis. Endothelial cells stimulated with conditioned medium from BMSCs treated with HG or HG + Bay. (e) and (f) Endothelial cell motility in each group was evaluated using the scratch wound assay. (g) and (h) Representative images and quantification of tube formation were assessed in each group. (i) and (j) Expression of Runx2 and VEGF protein in each group by western blot. Data are presented as the mean ± SD from at least three independent experiments. ^*∗*^*p* < 0.05 and ^*∗∗*^*p* < 0.01 versus HG group.

**Figure 6:** Cur prevented diabetes-induced bone loss and promoted vessel formation *in vivo*. (a) Experimental design illustrating the time points for inducing diabetes by STZ, establishing the DM model, and the timing of curcumin administration in the animal model. (b)–(g) Micro-CT images and (b) quantitative CT analysis (c)–(g) were performed in the distal femur from normal mice, DM mice, and DM mice treated with Cur. (h) Images of microfil perfusion. (i) Representative immunostaining images for CD31 (green) and EMCN (red) in the distal femur. (j) The Emcn^hi^ CD31^hi^ (yellow) cells were quantified. Data are shown as mean ± SD. ^*∗*^*p* < 0.05 and ^*∗∗*^*p* < 0.01 versus CON group. ^#^*p* < 0.05 and ^##^*p* < 0.01 versus DOP group.

The article "Curcumin Prevents Diabetic Osteoporosis through Promoting Osteogenesis and Angiogenesis Coupling via NF-κB Signaling" was published in 2022. Journal: Evid Based Complement Alternat Med.

## Data Availability

The data used to support the findings of this study are included within the article.
